RETRACTED

# The Analysis of Potential Diagnostic and Therapeutic Targets for the Occurrence and Development of Gastric Cancer Based on Bioinformatics

**DOI:** 10.1155/2022/4321466

**Published:** 2022-06-17

**Authors:** Chuan Ding, Qiqi Zhang, Xinying Jiang, Diandian Wei, Shu Xu, Qingdai Li, Meng Wu, Hongbin Wang

**Affiliations:** ^1^Department of Oncology, The Affiliated Hospital of Xuzhou Medical University, Xuzhou, Jiangsu 221000, China; ^2^Department of Laboratory, The Affiliated Hospital of Xuzhou Medical University, Xuzhou, Jiangsu 221000, China; ^3^Department of Oncology, Affiliated Hospital of Nantong University, Nantong, Jiangsu 226000, China

## Abstract

**Objective:**

Gastric cancer is among the most common malignant tumors of the digestive system. This study explored the molecular mechanisms and potential therapeutic targets for gastric cancer occurrence and progression using bioinformatics.

**Methods:**

The gastric cancer microarray dataset was downloaded from the Gene Expression Omnibus (GEO) database. The R package was used for data mining and screening differentially expressed genes (DEGs). Gene Ontology (GO) analysis and Kyoto Encyclopedia of Gene and Genome (KEGG) pathway analysis were performed using the Database for Annotation, Visualization, and Integrated Discovery (DAVID). Based on the protein-protein interaction (PPI) network analysis, core targets and core subsets were screened. Then, the relationship between the expression level of the core genes and the prognosis of gastric cancer patients was analyzed using the Gene Expression Profiling Interactive Analysis (GEPIA) database.

**Results:**

Using the GSE19826 and GSE54129 datasets, a total of 550 DEGs were identified, including 248 upregulated and 302 downregulated genes. GO and KEGG analyses showed that the upregulated DEGs were mainly enriched in the extracellular matrix (ECM) organization of the biological process (BP), the collagen-containing ECM of cellular component (CC), and the ECM structural constituent of molecular function (MF). DEGs were also enriched in human papillomavirus infections, the focal adhesion pathway, PI3K-Akt signaling pathway, and among others. The downregulated DEGs were mainly enriched in digestion, basal part of the cell, and aldo-keto reductase (NADP) activity. And the above pathways were enriched primarily in the metabolism of xenobiotics by cytochrome P450, drug metabolism-cytochrome P450, and retinol metabolism. Five core genes, including COL1A2, COL3A1, BGN, FN1, and VCAN, were significantly highly expressed in gastric cancer patients and were associated with poor prognosis.

**Conclusion:**

This study identified new potential molecular targets closely related to gastric cancer occurrence and development via mining public data using bioinformatics analysis methods.

RETRACTED

## 1. Introduction

Gastric cancer is the fifth most common malignant tumor and the fourth leading cause of cancer-related death worldwide, after lung cancer, colorectal cancer, and liver cancer [1]. According to the statistics of 2020 Global Cancer, about 1.09 million new gastric cancer cases and 769,000 gastric cancer death cases occurred globally in 2020 [1]. In China, gastric cancer is ranked third in incidence and mortality [2]. Although the incidence of gastric cancer has steadily declined in many countries, a trend whereby more and more younger people are being diagnosed with gastric cancer has been observed and cannot be ignored [3, 4]. Current treatments for gastric cancer include multimodal treatment using a combination of surgery, chemotherapy, radiotherapy, and/or immunotherapy [5–7]. Due to the asymptomatic and insidious nature, gastric cancer is rarely diagnosed in its early stage in China, and most patients have already advanced disease stage by the time of diagnosis and have poor prognoses [8–10]. Thus, the early detection and treatment of gastric cancer are crucial to improving treatment outcomes, and reducing its mortality rate is essential.

The rapid development of gene chip high-throughput sequencing technology has accumulated much disease-related data since the past ten years. This has led to the establishment of public databases, which have become an essential resource for scientific research, such as disease pathogenesis exploration and therapeutic target discovery [11]. Bioinformatics data mining of gene expression profiles using the Gene Expression Omnibus (GEO) database has led to identifying promising biomarkers associated with disease development [12]. At present, gene chip technology has a vital role in diagnosing gastric cancer and evaluating related gene expression [13]. In this study, a data mining strategy was used to obtain 2 microarray datasets of gastric cancer from the GEO database to identify differentially expressed genes (DEGs) associated with gastric cancer occurrence and progression. Then, a protein-protein interaction network (PPI) related to gastric cancer was constructed by Gene Ontology (GO) and Kyoto Encyclopedia of Genes and Genomes (KEGG) analyses, and the relationship of selected key genes with the survival of gastric cancer using Gene Expression Profile Interaction Analysis (GEPIA) was assessed. Overall, this study explored differential expressed genes (DEGs) associated with the occurrence and progression of gastric cancer and assessed their significance in the survival of gastric cancer to identify new diagnostic markers and potential therapeutic targets for gastric cancer.

RETRACTED

## 2. Materials and Methods

### 2.1. Data Collection

Gastric cancer gene expression profiling data (GSE19826 and GSE54129) were downloaded from the GEO database. The selection criteria for the above two gene expression profiles were as follows: (1) The included datasets must have contained data on paired gastric cancer and normal control tissues; (2) Both gene expression profiles were from the GPL570 (hg-u133_plus_2) Affymetrix Human Genome U133 Plus 2.0 Array. The flowchart of the data analysis of this study is shown in Figure 1.

### 2.2. Identification of DEGs

The data were read using the R language package, and each dataset was normalized using the limma R package [14]. All gene expression data were transformed via log2. The Fragments Per Kilobase Million (FPKM) value was applied to calculate the difference in gene expression between cancer tissues and adjacent tissues, and the *t*-test was used to analyze the significance of gene expression differences. The ∣logFC | >1 and *p* value < 0.05 were considered as the cut-off condition for screening DEGs between gastric cancer tissues and normal adjacent tissues.

### 2.3. GO and KEGG Enrichment Analyses of DEGs

Database for Annotation, Visualization, and Integrated Discovery (DAVID) (https://david.ncifcrf.gov/) was used to analyze the enrichment of GO and KEGG pathways of DEGs [15]. The GO knowledgebase is the world's largest source of information on the functions of genes and includes the following 3 domains: biological process (BP), cellular component (CC), and molecular function (MF). GO was used to identify those BP, cellular locations, and MF of the DEGs of interests. KEGG is a knowledgebase for the systematic analysis of gene functions, linking genomic information with higher order functional information. It consists of the PATHWAY, GENES, and LIGAND databases. It was used to determine the involvement of target genes in different biological. *P* < 0.05 was considered statistically significant.

### 2.4. Protein-Protein Interaction (PPI) Network Analysis and Core Gene Screening

PPI analysis was used to examine the interaction between genes that could be associated with gastric cancer occurrence and progression and could provide information for improving the diagnosis and treatment of these patients. The STRING database (http://string-db.org) was used to identify PPI between overlapping DEGs [16]. PPI networks were visualized and analyzed using Cytoscape 3.8.0 [17]. The core genes of the differential gene PPI networks were screened using the Maximal Clique Centrality (MCC) topology algorithm in the CytoHubb module in the Cytoscape plug-in. The module in the Hub web block was captured by the Cytoscape plug-in Molecular Complex Detection (MCODE).

RETRACTED

### 2.5. Statistics and Survival Analysis of Key Genes

The Gene Expression Profiling Interactive Analysis (GEPIA) website (http://gepia2.cancer-pku.cn/#index) was adopted for survival analysis of the expression of key genes in gastric cancer. The upper and lower 50% of gene expression was utilized as the analysis standard, and the Log-rank test for *P* < 0.05 was considered statistically significant.

## 3. Results

### 3.1. DEG Screening

In this study, two microarray datasets (GSE19826 and GSE54129) of gastric cancer were analyzed, and the information is shown in Table 1. The GSE19826 database contained 12 tumor and 15 normal tissues, while the GSE54129 database contained 111 tumor and 21 normal tissues. Additionally, 1934 DEGs were screened from the GSE19826 dataset, including 942 upregulated and 992 downregulated genes. From the GSE54129 dataset, 2503 DEGs were screened, including 1230 upregulated and 1273 downregulated genes. The cluster heat maps of DEGs are shown in Figures 2(a) and 2(b).

The top green bars represent gastric cancer tissues, and the orange bars represent normal gastric tissues. In the heat map, a greater red color intensity represents a higher gene expression level, while a greater blue color intensity represents a lower gene expression level.

### 3.2. GO and KEGG Analyses of DEGs

Collection of the differential genes of the two datasets using Venny 2.1.0 revealed the appearance of 550 DEGs on both chips. In all, 248 genes were upregulated, and 302 were downregulated (Figures 3(a) and 3(b)). GO functional annotation and KEGG pathway enrichment analysis of shared DEGs were performed using DAVID. The GO results showed (Figures 3(c) and 3(d)) that the upregulated DEGs were mainly enriched in the ECM organization of BP, the collagen-containing ECM of CC, and the ECM structural constituent of MF. Further, the downregulated DEGs were mainly enriched in digestion, basal part of the cell, and aldo-keto reductase (NADP) activity. KEGG analysis showed that the upregulated DEGs were mainly enriched in human papillomavirus infection, the focal adhesion pathway, PI3K-Akt signaling pathway, and other pathways. The downregulated DEGs were primarily enriched in pathways such as metabolism of xenobiotics by cytochrome P450 (CYPs), drug metabolism-CYPs, retinol metabolism, and other pathways (Figures 3(e) and 3(f)).

### 3.3. Differential Gene PPI Network Analysis

A total of 550 shared differential genes were submitted to the STRING 11.0 database by the Cytoscape 3.8.0 software, and the PPI network diagram was obtained (Figure 4(a)). According to the core genes screened by the MCC algorithm, the top 10 genes included were COL1A1, COL1A2, COL3A1, COL5A1, BGN, COL6A3, FN1, COL11A1, COL6A2, and COL4A2 (Figure 4(b)). In addition, according to the module analysis of the MCODE plug-in, a score > 5 points was considered the core subset. In this study, the core genes in the three core subnets were found to be COL11A1, GKN1, and VCAN (Figures 4(c)–4(e)).

RETRACTED

### 3.4. Expression Analysis of Core Genes in Gastric Cancer

The TCGA database was used to analyze the expression of 12 core genes, including COL1A1, COL1A2, COL3A1, COL5A1, BGN, COL6A3, FN1, COL11A1, COL6A2, COL4A2, GKN1, and VCAN in gastric cancer patients. The analysis results are shown in Figure 5, from which we found that except for GKN1, the other 11 core genes were highly expressed in gastric cancer patients. Among them, except for COL6A2, the expression levels of the remaining 10 core genes in gastric cancer tissues were significantly different from those in normal tissues (*P* < 0.05). For GKN1, the expression level in gastric cancer tissues was significantly decreased (*P* < 0.05).

### 3.5. Relationship between Core Genes and Survival Prognosis of Gastric Cancer Patients

The relationship between the 12 core genes and the survival of gastric cancer patients was analyzed using the GEPIA database. The analysis results showed that among the 12 core genes, the expression of COL1A2, COL3A1, BGN, FN1, and VCAN was significantly associated with the survival of gastric cancer patients (*P* < 0.05) (Figures 6(a)–6(l)). Lower expression of these genes was associated with higher survival rates.

## 4. Discussion

In this study, a total of 550 DEGs were identified by assessing the GSE19826 and GSE54129 datasets, of which 248 genes were upregulated, and 302 were downregulated in gastric cancer compared to normal tissues. Specifically, GO analysis showed that the upregulated DEGs were mainly enriched in the ECM organization of BP, the collagen-containing ECM of CC, and the ECM structural constituent of MF. The downregulated DEGs were mainly enriched in the digestion of BP, the basal part of the cell of CC, and the aldo-keto reductase (NADP) activity of MF.

The ECM regulates cell and tissue development and functions [18]. Their composition acts with specificity in different types of tissues, and highly distinctive ECMs can be found in different parts of the body. As such, the production and assembly of the ECM are an important aspect of maintaining cell and tissue homeostasis, and disruptions of the relative abundance of ECM proteins or their interactions with one another could lead to pathological conditions such as cancer [19, 20]. Studies have found that the ECM in solid tumors differs significantly from normal tissues and was associated with malignancy, tumor growth, and their response to treatment [21]. The effect of ECM on gastric cancer has been demonstrated in all steps, that is, from the degradation of the ECM, epithelial-to-mesenchymal transition (EMT), tumor angiogenesis, development of an inflammatory tumor microenvironment, to cancer metastasis [22]. In a study by Tiitta et al. [23], the authors found that invading diffuse gastric cancer had no tenascin (Tn) in their submucosa and muscle cell layers while invading intestinal type gastric cancer islets had prominent expression of Tn. They concluded that Tn is an important stromal component in malignant growth and in lesions undergoing active repair and remodelling. Generally, abnormal collagen expression usually appears in gastric cancer tissues, and their level varies between premalignant and malignant lesions. By comparing the stomach tissues of individuals with normal, premalignant, and malignant lesions, Zhao et al. found that some collagen genes, such as COL4A1 and COL5A1, were significantly increased in malignant lesions of stomach compared with in premalignant lesions and were independent prognostic markers [24]. Further, ECM characterization in gastric cancer has been shown to predict treatment response and prognosis [25]. Thus, as more experimental and clinical observations are strongly indicating that ECM constituents, receptors and associated signaling molecules are promising biomarkers of prognosis and/or therapeutic targets; novel and more effective gastric cancer treatments that combine strategies targeting ECM with corresponding inhibitors or immuno-oncology agents could lead to improve therapeutic outcomes.

RETRACTED

KEGG enrichment analysis revealed that upregulated DEGs were mainly enriched in human papillomavirus (HPV) infection, the focal adhesion pathway, PI3K-Akt signaling pathway, and other pathways. The downregulated DEGs were mainly enriched in the metabolism of xenobiotics by CYPs, drug metabolism-CYPs, and retinol metabolism. Through a meta-analysis, Zeng et al. [26] pointed out that HPV may be a potential risk factor for gastric cancer. They also observed that the HPV prevalence was reported to be much more common in oral and anal cancers (58.0% and 80%) than in gastric cancer, suggesting that the route of HPV entering the body could be associated with the risk of HPV-related cancers. In regard to gastric cancer, it is assumed that the infection could enter from the mouth and descends to the stomach. Persistent HPV infection and associated injury could lead to dysplasia or adenocarcinoma in situ, resulting in malignant transformation. It was even reported that coinfection with Helicobacter pylori could also lead to canceration [27], although such an argument remains controversial [28]. Park et al. [29] reported that, in gastric cancer patients, the protein expression of focal adhesion kinase (FAK) was positively correlated with tumor size, depth of tumor invasion, lymph node metastasis, distant metastasis, lymphatic invasion, and venous invasion. Focal FAK gene amplification was positively associated with age, tumor size, lymph node metastasis, distant metastasis, lymphatic invasion, venous invasion, and perineural invasion. FAK protein expression or gene amplification was significantly correlated with tumor progression and poor prognosis in gastric cancer. Ying et al. [30] found that the positive expression rates of PI3K, p-AKT, and p-mTOR in gastric cancer were 49%, 58%, and 56%, respectively, and gastric cancer patients with PI3K/p-AKT/p-mTOR had a poor prognosis. The roles of CYPs are mainly focused on the studies of hepatic drug metabolism, cardio physiology, and hypertension. According to data from earlier studies, the expression of CYP1A and CYP3A proteins was detected in 51% and 28% of gastric cancer cases, respectively, but not in normal gastric tissue [31]. Recent studies have shown that elevated expression of CYP3A4 may be associated with the progression of chronic atrophic gastritis to gastric cancer [32]. Overexpression of CYP2E1 can activate the PI3K-AKT-mTOR signaling pathway in gastric cancer cells [32]. Overall, few studies have been conducted on intragastric CYPs, possibly because the expression of CYPs is generally lower in the normal gastric mucosa than in other parts of the gastrointestinal tract, and the role of CYPs in driving gastric carcinogenesis remains largely unknown. Also, more studies are needed to understand the potential significance of CYPs in gastric cancer [33].

Expression and prognosis analysis showed that the expression level of 12 core genes was significantly changed in gastric cancer compared with normal gastric tissues. Five genes, including COL1A2, COL3A1, BGN, FN1, and VCAN, were notably correlated with the survival and prognosis of gastric cancer patients. When the expression level of the above genes was low, the survival rate of patients was high. COL1A2 and COL3A1 encode the pro-*α*2 chain of type I collagen and the pro-*α*1 chain of type III collagen, respectively. Collagen is a major structural component of the ECM, providing tensile strength, regulating cell adhesion, supporting chemotaxis and migration, and directly regulating development. Studies have revealed that collagen genes are closely related to the occurrence and development of tumors, which are gradually considered effective for tumor diagnosis and prognosis. Using data mining methods, Hu et al. [34] also found a significant upregulation in COL1A1, COL1A2, COL6A3, and SULF1 genes in gastric adenocarcinoma and a notable correlation between the above genes and TNM staging. Zhuo et al. [35] found that multiple genes, including COL1A2, were expressed at a high level in gastric cancer tissues. Li et al. [36] found that a high mRNA expression level of COL1A2 was positively correlated with tumor size and depth of invasion, which may predict poor clinical prognosis in gastric cancer patients. In addition to gastric cancer, research reports from different teams have shown that multiple collagen-encoding genes, including COL1A2 and COL3A1, have higher expression level in pancreatic cancer [37], thyroid cancer [38], esophageal cancer [39], and others. The above genes have been shown to regulate the proliferation, migration, and invasion of cancer cells. Biglycan is encoded by the BGN gene, a key member of the small leucine-rich proteoglycans family, is an important component of the ECM. Clinical studies have shown that the upregulation of BGN is associated with poor prognosis in patients with various solid tumors. Studies have found that the mRNA expression level of BGN is increased in bladder, brain, central nervous system, breast, colorectal, esophageal, gastric, head and neck, and lung and ovarian cancer, including 28 subtypes of cancers compared with normal tissues. Their increased expression is thought to be associated with poor prognosis in ovarian and gastric cancers [40]. The experimental study results of Hu et al. [41] indicated that BGN induced increased phosphorylation levels in FAK (Tyr576/577, Tyr925, and Tyr397) and paxillin and enhanced the wound healing, migration, and invasion abilities of gastric cancer cells, as well as the tube formation ability of endothelial cells. Besides, BGN was correlated with lymph node metastasis, depth of tumor invasion, and tumor-node-metastasis (TNM) stage. Fibronectin encoded by the FN1 gene is a glycoprotein and a major component of the ECM. Besides, fibronectin regulates the proliferation, motility behavior, and fate of multiple cell types through integrin-mediated signal transduction mechanisms. For one thing, fibronectin is expressed widely in human cancers as a large multidomain glycoprotein dimer. For another, fibronectin can utilize cell-driven forces to assemble into a fibrous array, providing a specialized stent and a binding site of soluble factor functionalization in the tumor microenvironment for the deposition of other matrix proteins [42, 43]. Studies have found that low FN1 expression was associated with prolonged survival in diffuse, poorly differentiated, and node-positive gastric cancer [44, 45]. Further, the expression level of FN1 has also been shown to be abnormally elevated in ovarian cancer [46], nasopharyngeal carcinoma [47], and other tumors and is considered a marker of poor prognosis. Versican is encoded by the VCAN gene and is not only a large chondroitin sulfate proteoglycan but also a major component of the ECM. Additionally, versican is involved in cell adhesion, proliferation, migration, and angiogenesis and plays a central role in tissue morphogenesis and maintenance [48]. Studies have reported that versican regulates tumor migration and invasion, and elevated versican expression was significantly associated with renal cancer metastasis and a poor 5-year overall survival rate in these patients even after radical nephrectomy [49]. Asano et al. [50] found that versican could regulate angiogenesis and promote tumor growth.

RETRACTED

Despite the promising findings observed from this study, there were some limitations that should be taken into consideration. First, the sample size used in this experiment could limit the generalization of the study conclusion, and further assessment in larger cohort and different populations would provide more robust evidence. Second, this study mainly utilized retrospective transcriptome analysis data and lacked validation. Therefore, *in vitro*, *in vivo*, and prospective data still need to be collected to validate the real-world clinical significance of the identified DEGs and core genes in relation to the occurrence, progression, and prognosis of gastric cancer. Lastly, more experiments are needed to clarify the upstream regulatory pathways and downstream mechanisms of the identified key differential genes.

## 5. Conclusion

This study assessed genes that were differently expressed between gastric cancer and normal gastric tissues. Compared to normal gastric tissues, 10 core genes, namely, COL1A1, COL1A2, COL3A1, COL5A1, BGN, COL6A3, FN1, COL11A1, COL4A2, and VCAN, were highly expressed in gastric cancer tissues while the expression of GKN1 was significantly decreased. Of them, higher expression of COL1A2, COL3A1, BGN, FN1, and VCAN was associated with poor survival. Further, upregulated DEGs were mainly enriched in the ECM organization of BP, the collagen-containing ECM of CC, and the ECM structural constituent of MF, and targeting the PI3K-Akt signaling pathway could be a promising strategy to improve treatment outcomes. However, further studies are needed to validate these findings.

## Figures and Tables

**Figure 1:** Flowchart of data analysis.

RETRACTED

**Figure 2:** Cluster heat map of differential genes of the (a) GSE19826 and (b) GSE54129 datasets.

**Figure 3:** GO analysis and KEGG analysis. (a, b) Venn diagram revealing the (a) upregulated differentially expressed genes and (b) downregulated differentially expressed genes shared in the GSE19826 and GSE54129 datasets. (c, d) GO analysis of shared (c) upregulated genes and (d) downregulated genes. (e, f) KEGG pathway enrichment analysis of commonly upregulated genes and (f) downregulated genes.

**Figure 4:** PPI network analysis: (a) PPI network diagram of shared differential genes; (b) core targets; (c–e) core subnets with a score > 5 based on MCODE. The squares represent the core genes in each subnet.

**Figure 5:** Expression level of the 12 core genes, including COL1A1, in gastric cancer tissues.

**Figure 6:** Core genes associated with the survival of gastric cancer patients: (a) COL1A1; (b) COL1A2; (c) COL3A1; (d) COL5A1; (e) BGN; (f) COL6A3; (g) FN1; (h) COL11A1; (i) COL6A2; (j) COL4A2; (k) GKN1; (l) VCAN.

**Table 1:** Basic information of the GEO datasets.

Datasets	Number of samples	Grouping	GPL information	Sample type
GSE19826	27	Gastric cancer tissues 12 cases, normal gastric tissue 15 cases	GPL570	mRNA
GSE54129	132	Gastric cancer tissues 111 cases, normal gastric tissue 21 cases	GPL570	mRNA

## Data Availability

The data used to support the findings of this study are available from the corresponding author upon request.
